RETRACTED

# Downregulation of microRNA-218 is cardioprotective against cardiac fibrosis and cardiac function impairment in myocardial infarction by binding to MITF

**DOI:** 10.18632/aging.102112

**Published:** 2019-08-13

**Authors:** Linfeng Qian, Shaobo Pan, Liping Shi, Yongyi Zhou, Lai Sun, Zhedong Wan, Yufang Ding, Jia Qian

**Affiliations:** 1 Department of Cardiothoracic Surgery, First Affiliated Hospital of Zhejiang University, Hangzhou 310003, PR. China; 2 Operating Room, First Affiliated Hospital of Zhejiang University, Hangzhou 310003, PR. China

**Keywords:** myocardial infarction, microRNA-218, microphthalmia-associated transcription factor, cardiac fibrosis, cardiomyocyte apoptosis

## Abstract

Objective: This study is intended to figure out the function of microRNA-218 (miR-218) together with microphthalmia-associated transcription factor (MITF) on the cardiac fibrosis and cardiac function impairment in rat models of myocardial infarction (MI).

Results: The rats with MI exhibited cardiac function impairment, cardiac fibrosis, oxidative stress, cardiomyocyte apoptosis, as well as inflammatory injury. Additionally, upregulated miR-218 and downregulated MITF were detected in cardiac tissues of MI rats. MI rats injected with miR-218 inhibitors or overexpressed MITF exhibited elevated MITF expression, improved cardiac function, and diminished pathological damages, infarct size, cardiomyocyte apoptosis, cardiac fibrosis, oxidative stress as well as inflammatory injury in cardiac tissues. Furthermore, downregulated miR-218 and MITF aggravated the conditions than downregulation of miR-218 alone in MI rats.

Methods: MI models were performed in rats, and then the rats were injected with miR-218 inhibitors and/or MITF overexpression plasmid to elucidate the role of miR-218 and/or MITF on the cardiac function, pathological damage, cardiac fibrosis, angiogenesis, oxidative stress and inflammatory injury of cardiac tissues in MI rats by performing a series of assays.

Conclusion: Collectively, we found that the suppression of miR-218 alleviates cardiac fibrosis and cardiac function impairment, and stimulates angiogenesis in MI rats through inhibiting MITF.

## INTRODUCTION

Myocardial infarction (MI) is a common deadly cardiovascular disease, and the damage caused by MI to cardiac tissues is likely to result in the occurrence of heart failure [1, 2]. In the settings of MI, the cardiomyocyte apoptosis or necrosis develops to disappearance of cardiomyocytes, which diminishes pumping of the heart and further leads to congestive heart failure [3, 4]. Cardiac fibrosis following MI can be observed in both the infarcted and non-infarcted myocardium, and excessive cardiac fibrosis progressively damages cardiac function and is involved with increased hospitalization and death rate related with heart failure [5]. Furthermore, angiogenesis plays a significant role in the cardiac repair, and suppressed angiogenesis may damage the cardiac repair and result in cardiac rupture [6]. It is urgent to identify new approaches to facilitate the hemodynamic function after MI for the proarrhythmogenic risks in patients with heart failure [7]. Accumulating studies have proposed microRNAs (miRs) as potential biomarkers in the treatment and prognosis of MI [8–10].

RETRACTED

MiRs are small non-coding RNAs which can mediate the gene expression at post-transcriptional level through translational repression or degradation of target mRNAs [11]. Multiple studies have reported a pivotal role for miR-dependent modulation of cardiac fibrosis, angiogenesis and cardiomyocyte hypertrophy following MI [12–14]. MicroRNA-218 (miR-218) has been recognized as a vertebrate-specific miR playing a critical role in tumorigenesis and progression through mediating the expression of target genes [15]. Previous studies have highlighted the tumor suppressor role of miR-218 in non-small cell lung cancer [16], pancreatic cancer [17] and gastrointestinal stromal tumors [18]. In the experimental model of zebrafish embryo development, miR-218 can affect cardiac development through circulatory regulation with Tbx5a, and inhibition of miR-218 can attenuate cardiac cycle insufficiency in embryonic heart development caused by overexpression of Tbx5a, while overexpression miR-218 can cause cardiac malformation, atrial hypoplasia, and ventricular septum insufficiency of zebrafish embryo [19]. Overexpression of miR-218 in zebrafish embryos can inhibit the normal development of heart [20, 21]. Overexpression of miR-218 can also inhibit the differentiation of mouse embryonic stem cells into mesoderm and cardiomyocytes [22]. Therefore, we speculate that miR-218 is associated with MI. Godwin et al. [23] used miRs microarray analysis to analyze miRs after renal ischemia-reperfusion injury in C57BL/6 mice, and found that the expression of miR-218 increased. Therefore, we hypothesized that miR-218 is highly expressed in MI. In this study, the targeting relationship between miR-218 and microphthalmia-associated transcription factor (MITF) is determined by bioinformatics prediction and a confirmatory dual-luciferase reporter gene assay. MITF mediates the development and differentiation of retinal pigment epithelium and melanocytes [24]. Interestingly, MITF has been documented as the target genes of miR-340 involved in osteoclast differentiation [25], and furthermore, MITF indirectly drives the expression of miR-211 by transcriptionally up-regulating transient receptor potential melastatin 1 (TRPM1) [26]. Notably, miR-218 represses melanogenesis via directly inhibiting the expression of MITF [27]. Hu et al. have found that miR-218 exerts functions in the transformation of hematopoietic cells via regulating the MITF pathway [28]. Therefore, in this study, we examined the expression of miR-218 and MITF in MI. Additionally, the effect of miR-218 and MITF on the cardiac fibrosis, cardiomyocyte apoptosis, angiogenesis, oxidative stress and inflammatory injury in rat models of MI was also investigated.

RETRACTED

## RESULTS

### MiR-218 is highly expressed in cardiac tissues and downregulated miR-218 improves cardiac function in MI rats

RT-qPCR was employed to determine the expression of miR-218 in cardiac tissues. Relative to the sham group, rats in the MI group showed increased miR-218 expression in cardiac tissues (*P* < 0.05) (Figure 1A), preliminarily suggesting the correlation of miR-218 with the occurrence of MI.

**Figure 1:** **MiR-218 is highly expressed in cardiac tissues and downregulated miR-218 improved cardiac function in MI rats.** (**A**) miR-218 expression in cardiac tissues of rats in the sham group and MI group detected by RT-qPCR, n = 3; (**B**) miR-218 expression in cardiac tissues of MI rats of the MI group, the MI + inhibitors NC group and the MI + miR-218 inhibitors group, n = 3; (**C**) the LVEF and LVFS of rats detected by ultrasonic cardiogram, n = 12; (**D**) the LVSP, LVEDP, +dp/dt max and -dp/dt max of rats detected by hemodynamic monitoring, n = 12; *versus the sham group, *P* < 0.05; #versus the MI group, *P* < 0.05; Data were analyzed by *t* test or one-way ANOVA. Pairwise comparison after ANOVA was performed by LSD-t. MI, myocardial infarction; miR-218, microRNA-218; LVEF, left ventricular ejection fraction; LVFS, left ventricular fraction shortening; LVSP, left ventricular systolic pressure; LVEDP, left ventricular end diastolic pressure; RT-qPCR, reverse transcription quantitative polymerase chain reaction.

Additionally, among the MI rats, the cardiac tissues of the MI + miR-218 inhibitors group had significantly lower miR-218 expression than the MI group and the MI + inhibitors NC group (both *P* < 0.05) (Figure 1B). This indicated that miR-218 inhibitors effectively suppressed the miR-218 expression in cardiac tissues of MI rats.

Ultrasonic cardiogram demonstrated that, compared with the sham group, there showed decreased cardiac function in the MI, MI + inhibitors NC and MI + miR-218 inhibitors groups, which was presented with reduced LVEF and LVFS (all *P* < 0.05). The MI + miR-218 inhibitors group had increased LVEF and LVFS relative to the MI and MI + inhibitors NC groups (both *P* < 0.05) (Figure 1C).

RETRACTED

The hemodynamic monitoring manifested that MI rats had higher LVEDP and lower LVSP, +dp/dt max and -dp/dt max than rats in the sham group (all *P* < 0.05). Relative to the MI and MI + inhibitors NC groups, the MI + miR-218 inhibitors group displayed reduced LVEDP and increased LVSP, +dp/dt max and -dp/dt max (all *P* < 0.05) (Figure 1D).

### Downregulated miR-218 alleviates pathological damage of cardiac tissues in rats with MI

The ratio of heart to body weight was higher in the MI and MI + inhibitors NC groups than that in the sham group, while the MI + miR-218 inhibitors group had lower ratio of heart to body weight than the MI and MI + inhibitors NC groups (all *P* < 0.05) (Figure 2A).

**Figure 2:** **Downregulated miR-218 expression alleviates pathological damage of cardiac tissues in MI rat models.** (**A**) the ratio of heart to body weight, n = 6; (**B**) serum levels of LDH and CPK examined by the biochemical analyzer, n = 6; (**C**) HE staining showing pathological changes of cardiac tissues (× 200), n = 3; (**D**) ultrastructure of cardiomyocytes observed by transmission electron microscope (× 5000), n = 3; (**E**) TTC staining showing the infarct size of rats, n = 3; (**F**) TUNEL staining showing the apoptotic index of cardiomyocytes (× 400), n = 3; (**G**) Western blot assay showing protein levels of apoptosis-related factors Bax and Bcl-2 in cardiac tissues, n = 3; *versus the sham group, *P* < 0.05; #versus the MI group, *P* < 0.05; Data were analyzed by one-way ANOVA. Pairwise comparison after ANOVA was performed by LSD-t. MI, myocardial infarction; miR-218, microRNA-218; LDH, lactate dehydrogenase; CPK, creatine phosphokinase.

The serum levels of LDH and CPK were examined by the biochemical analyzer. Relative to the sham group, the MI rats showed significantly increased serum levels of LDH and CPK. After the treatment of miR-218 inhibitors, the serum levels of LDH and CPK were obviously decreased (*P* < 0.05) (Figure 2B).

HE staining was used to observe pathological changes of cardiac tissues. Rats in the sham group show no pathological changes in cardiac tissues, with evenly stained and aligned cardiomyocytes and uniform clear space between cardiomyocytes. In the MI and MI + inhibitors NC groups, we observed unevenly stained and aligned cardiomyocytes. The space between cardiomyocytes was narrowed and broken. Some dotted bleeding could be seen near the broken myocardium. We also found massive myocardial necrosis, with obvious inflammatory infiltration and severe fibrous connective tissue hyperplasia in the necrotic region. The MI + miR-218 inhibitors group showed slight pathological changes in cardiac tissues. The cardiomyocytes were basically evenly stained and aligned with normal appearance. The space between cardiomyocytes was also even. Meanwhile, the space between cardiomyocytes was narrowed and the myocardium was slightly enlarged. Little myocardial necrosis, slight inflammatory infiltration and fibrous connective tissue hyperplasia were also observed (Figure 2C).

RETRACTED

The TEM observation demonstrated that the cardiac tissues in the sham group displayed evenly aligned myofilaments, clear difference in sarcomere between light and dark and evenly aligned mitochondria along myofilaments. In the MI and MI + inhibitors NC groups, the myofilaments were broken, dissolved and loosely aligned. The mitochondria were unevenly aligned. Karyopyknosis and highly edema of cytoplasm around the nucleus were observed. In addition, in the MI + miR-218 inhibitors group, broken and dissolved myofilaments could be observed, but the difference in sarcomere between light and dark was clear, the mitochondria were evenly aligned and a few mitochondria were vacuolated (Figure 2D).

After TTC staining, we observed that the sham group showed no infarction and rats in the MI groups had MI formation. Massive MI was observed in the MI and MI + inhibitors NC groups. The treatment of miR-218 inhibitors reduced size of infarct in MI rats (*P* < 0.05) (Figure 2E).

TUNEL staining was employed to examine apoptosis of cardiomyocytes. Few Apoptotic cardiomyocytes were observed in the sham group. The MI and MI + inhibitors NC groups had higher apoptotic index of cardiomyocytes than the sham group and the MI + miR-218 inhibitors group (*P* < 0.05) (Figure 2F).

Western blot assay was performed to determine protein levels of apoptosis-related factors Bax and Bcl-2 in cardiac tissues. The protein level of Bax was increased and that of Bcl-2 was reduced in the MI and MI + inhibitors NC groups, relative to the sham group. The MI + miR-218 inhibitors group had lower protein level of Bax and higher protein level of Bcl-2 than MI and MI + inhibitors NC groups (all *P* < 0.05) (Figure 2G).

### Downregulated miR-218 reduces cardiac fibrosis and promotes angiogenesis in rats with MI

According to the evaluation of Masson staining, the sham group were presented with evenly aligned red cardiac tissues with little collagen tissues. In the MI and MI + inhibitors NC groups, cardiac tissues were replaced by collagen tissues, with few disorderly aligned cardiomyocytes possessing vague structure. The collagen in the cardiac tissues was higher in the MI and MI + inhibitors NC groups than the sham group. The MI + miR-218 inhibitors group mainly showed red cardiac tissues, mixed with collagen tissues. The cardiac tissues were relatively evenly aligned with some broken tissues, which were replaced by fibrous tissues. The collagen in the cardiac tissues was lower in the MI + miR-218 inhibitors group than the MI and MI + inhibitors NC groups (*P* < 0.05) (Figure 3A).

RETRACTED

**Figure 3:** **Downregulated miR-218 expression reduces cardiac fibrosis and promotes angiogenesis in MI rats.** (**A**) Masson staining showing the cardiac fibrosis of rats (× 200); (**B**) immunohistochemical staining showing the expression of type I collagen and type III collagen (× 200); (**C**) CD34 immunohistochemistry showing MVD and MMVD of cardiac tissues (× 200); (**D**) the mRNA expression of angiogenesis-related factor VEGF detected by RT-qPCR; (**E**) the protein expression of angiogenesis-related factor VEGF detected by western blot assay. *versus the sham group, *P* < 0.05; #versus the MI group, *P* < 0.05; n = 3. Data were analyzed by one-way ANOVA. Pairwise comparison after ANOVA was performed by Fisher’s least significant difference. MI, myocardial infarction; miR-218, microRNA-218; MVD, microvascular density; MMVD, mean microvessels diameter; RT-qPCR, reverse transcription quantitative polymerase chain reaction; VEGF, vascular endothelial growth factor.

Based on the immunohistochemical staining, the sham group didn’t show stained brown cells. The MI and MI + inhibitors NC groups showed massive stained brown cells. The quantitative analysis found that the MI and MI + inhibitors NC groups had higher expression of type I collagen and type III collagen than that in the sham group. The expression of type I collagen and type III collagen in the MI + miR-218 inhibitors group was lower than the MI and MI + inhibitors NC groups (all *P* < 0.05) (Figure 3B).

After MI, coronary artery occlusion together with myocardial ischemia and hypoxia result in loss of myocardial tissue, directly lead to myocardial tissue necrosis and apoptosis. The amount of angiogenesis after MI is closely related to the improvement of cardiac function and morphology after MI. CD34 immunohistochemistry was employed to examine the microvascular density (MVD) of cardiac tissues. MVD in the MI group was higher than that in the sham group. The MI + miR-218 inhibitors group showed increased MVD as compared with the MI and MI + inhibitors NC groups (*P* < 0.05). There was no significant difference in MVD between the MI and MI + inhibitors NC groups (*P* > 0.05). Meanwhile, mean microvessels diameter (MMVD) in the MI group was lower than that in the sham group. The MI + miR-218 inhibitors group showed increased MMVD as compared with the MI and MI + inhibitors NC groups (*P* < 0.05). There was no significant difference in MMVD between the MI and MI + inhibitors NC groups (*P* > 0.05) (Figure 3C).

RETRACTED

The mRNA and protein expression of angiogenesis-related factor VEGF was determined. After model establishment, the MI rat models displayed increased mRNA and protein expression of VEGF (*P* < 0.05). When the miR-218 expression was inhibited in MI rat models, the mRNA and protein expression of VEGF was increased (*P* < 0.05) (Figure 3D–3E).

### Downregulated miR-218 reduces oxidative stress and inflammatory injury in rats with MI

The spectrocolorimetric method was employed to evaluate the levels of malondialdehyde (MDA) in tissue homogenate and the activity of GSH-Px and SOD. After model establishment, MI rat models displayed obvious lipid peroxidation, presenting with increased serum levels of MDA and diminished activity of GSH-Px and SOD. The injection of miR-218 inhibitors through caudal vein downregulated the miR-218 expression, whereby the serum levels of MDA were diminished and activity of GSH-Px and SOD was promoted (all *P* < 0.05) (Figure 4A).

**Figure 4:** **Downregulated miR-218 expression reduces oxidative stress and inflammatory injury in MI rats.** (**A**) the levels of MDA and the activity of GSH-Px and SOD determined by the spectrocolorimetric method, n = 3; (**B**) the mRNA expression of IL-1β, IL-6 and TNF-α detected by RT-qPCR, n = 3; (**C**) the serum levels of IL-1β, IL-6 and TNF-α detected by ELISA, n = 6; *versus the sham group, *P* < 0.05; #versus the MI group, *P* < 0.05; Data were analyzed by one-way ANOVA. Pairwise comparison after ANOVA was performed by LSD-t. MI, myocardial infarction; miR-218, microRNA-218; ELISA, enzyme-linked immunosorbent assay; IL-1β, interleukin-1β; IL-6, interleukin-6; TNF-α, tumor necrosis factor-α; MDA, malondialdehyde; GSH-Px, glutathione peroxidase; SOD, superoxide dismutase; RT-qPCR, reverse transcription quantitative polymerase chain reaction.

Based on RT-qPCR analysis, relative to the sham group, the mRNA expression of IL-1β, IL-6 and TNF-α in cardiac tissues was elevated in the MI group. The MI group and the MI + inhibitors NC group didn’t differ significantly in mRNA expression of IL-1β, IL-6 and TNF-α in cardiac tissues (*P* > 0.05). Compared with the MI and MI + inhibitors NC groups, the MI + miR-218 inhibitors group had diminished mRNA expression of IL-1β, IL-6 and TNF-α in cardiac tissues (*P* < 0.05) (Figure 4B). ELISA was performed to determine the serum levels of IL-1β, IL-6 and TNF-α, and the tendencies were consistent with the RT-qPCR analysis (Figure 4C). These results suggested that inhibited miR-218 expression could alleviate the oxidative stress and inflammatory injury of MI rats.

RETRACTED

### MITF is a target gene of miR-218

According to the results of RT-qPCR and western blot assay, compared with the sham group, the mRNA and protein expression of MITF in the cardiac tissues of MI rats was reduced (*P* < 0.05). Versus the MI group, the MI + miR-218 inhibitors group showed increased mRNA and protein expression of MITF in the cardiac tissues of MI rats (*P* < 0.05). No significant difference was identified in the mRNA and protein expression of MITF between the MI and MI + inhibitors NC groups (*P* > 0.05) (Figure 5A–5B). These preliminarily indicated the MITF may participate in the occurrence of MI and miR-218 may be negatively correlated with MITF in MI.

**Figure 5:** **The targeting relationship between miR-218 and MITF is determined by bioinformatics prediction and a confirmatory dual-luciferase reporter gene assay.** (**A**) the mRNA expression of MITF detected by RT-qPCR; (**B**) the protein expression of MITF detected by western blot assay; (**C**) the binding sites of miR-218 to MITF predicted by online software; (**D**) the targeting relationship of miR-218 and MITF determined by dual-luciferase reporter gene assay; (**D**) * versus the sham group, *P* < 0.05; # versus the MI group, *P* < 0.05; n = 3. Data were analyzed by one-way ANOVA. Pairwise comparison after ANOVA was performed by LSD-t.

The targeting relationship of miR-218 to MITF was predicted by bioinformatics software (http://www.targetscan.org) (Figure 5C). The luciferase activity detection indicated that, compared with the co-transfection of MITF-3′UTR-MUT + mimics NC, the cells with co-transfection of MITF-3′UTR-WT and miR-218 mimics showed reduced luciferase activity (*P* < 0.01). Whereas, relative to the co-transfection of MITF-3′UTR-MUT and mimics NC, the cells with co-transfection of MITF-3′UTR-MUT and miR-218 mimics didn’t differ significantly (*P* > 0.05) (Figure 5D).

### Upregulated MITF improves cardiac function in rats with MI

The interference efficiency of MITF was assessed by RT-qPCR and western blot assay. The mRNA and protein expression of MITF in the cardiac tissues in the MI and MI + inhibitors NC groups wasn’t different (*P* > 0.05). Compared with the MI group, the MI + MITF group showed increased mRNA and protein expression of MITF in the cardiac tissues (*P* < 0.05) (Figure 6A–6B), suggesting that the interference of overexpressing MITF is successful.

**Figure 6:** **Upregulated MITF expression improves cardiac function in MI rats.** (**A**) the mRNA expression of MITF in cardiac tissues of MI rats detected by RT-qPCR, n = 3; (**B**) the protein expression of MITF in cardiac tissues of MI rats detected by western blot assay, n = 3; (**C**) the LVEF and LVFS of rats detected by ultrasonic cardiogram, n = 12; (**D**) the LVSP, LVEDP, +dp/dt max and -dp/dt max of rats detected by hemodynamic monitoring, n = 12; * versus the sham group, *P* < 0.05; # versus the MI group, *P* < 0.05; Data were analyzed by *t* test or one-way ANOVA. Pairwise comparison after ANOVA was performed by LSD-t. MI, myocardial infarction; LVEF, left ventricular ejection fraction; LVFS, left ventricular fraction shortening; LVSP, left ventricular systolic pressure; LVEDP, left ventricular end diastolic pressure; RT-qPCR, reverse transcription quantitative polymerase chain reaction; MITF, microphthalmia-associated transcription factor.

RETRACTED

According to the ultrasonic cardiogram, relative to the rats in the sham group, lower LVEF and LVFS were identified in the MI group and the MI + MITF-NC group, while higher LVEF and LVFS were identified in the MI + MITF group (*P* < 0.05) (Figure 6C).

Based on the hemodynamic monitoring, the MI group and the MI + MITF-NC group weren’t significantly different in the hemodynamic indicators (*P* > 0.05). The MI + MITF group displayed lower LVEDP and higher LVSP, +dp/dt max and -dp/dt max than the MI group (all *P* < 0.05) (Figure 6D).

### Upregulated MITF alleviates pathological damage of cardiac tissues in rats with MI

The ratio of heart to body weight was higher in the MI and MI + MITF-NC groups than that in the sham group. Upregulation of MITF could decrease the ratio of heart to body weight of MI rats (*P* < 0.05) (Figure 7A).

**Figure 7:** **Upregulated MITF expression alleviates pathological damage of cardiac tissues in MI rats.** (**A**) the ratio of heart to body weight, n = 6; (**B**) serum levels of LDH and CPK examined by the biochemical analyzer, n = 6; (**C**) HE staining showing pathological changes of cardiac tissues (× 200), n = 3; (**D**) ultrastructure of cardiomyocytes observed by transmission electron microscope (× 5000), n = 3; (**E**) TTC staining showing the infarct size of rats, n = 3; (**F**) TUNEL staining showing the apoptotic index of cardiomyocytes (× 400), n = 3; (**G**) Western blot assay showing protein levels of apoptosis-related factors Bax and Bcl-2 in cardiac tissues, n = 3; * versus the sham group, *P* < 0.05; # versus the MI group, *P* < 0.05; Data were analyzed by one-way ANOVA. Pairwise comparison after ANOVA was performed by LSD-t. MI, myocardial infarction; MITF, microphthalmia-associated transcription factor; LDH, lactate dehydrogenase; CPK, creatine phosphokinase.

The biochemical analysis indicated that compared with the MI and MI + MITF-NC groups, the serum levels of LDH and CPK were higher than those in the sham group and the MI + MITF group (*P* < 0.05) (Figure 7B).

RETRACTED

The results of HE staining manifested that, in the sham group, the cardiomyocytes were uniformly and densely arranged with clear structure. Not much extracellular matrix and a few fibroblasts were observed. In the MI and MI + MITF-NC groups, the cardiomyocytes were weakly stained with disorder arrangement, vague structure, karyolysis, reduction of nuclei and even disappearance of nuclei. Increased fibroblasts and obvious inflammatory infiltration were observed. In the MI + MITF group, the nuclei of cardiomyocytes were enlarged and the cell structure was slightly vague. Slight hyperplasia of fibroblasts and a little inflammatory infiltration was observed (Figure 7C).

The TEM observation demonstrated that cardiomyocytes in the sham group had normal ultrastructures. The cardiomyocytes in the MI and MI + MITF-NC groups were weakly stained. The majority of myofibrils were broken or disappeared. The mitochondria and granular endoplasmic reticulum were reduced. Mitochondria were vacuolated, with most mitochondrial membrane and cristae broken or disappeared. The MI + MITF group showed mild edema around the nucleus. The mitochondria displayed mild edema, with some broken membrane and cristae (Figure 7D).

The analysis of TTC staining suggested that the MI + MITF group showed smaller infarct size than the MI and MI + MITF-NC groups (*P* < 0.05) (Figure 7E).

The results of TUNEL staining indicated that the apoptotic index of cardiomyocytes between the MI group and the MI + MITF-NC group weren’t significantly different (*P* > 0.05). Compared with the MI and MI + MITF-NC groups, the MI + MITF group showed inhibited apoptotic index of cardiomyocytes (*P* < 0.05) (Figure 7F).

According to the results of western blot assay, the protein level of Bax was increased and that of Bcl-2 was reduced in the MI rats. The upregulation of MITF decreased the protein level of Bax and promoted the protein level of Bcl-2 (*P* < 0.05) (Figure 7G).

### Upregulated MITF inhibits cardiac fibrosis and promotes angiogenesis in rats with MI

According to the Masson staining, we found that rats in the sham group were mainly red myocardial tissue, collagen tissue distribution was rare, and myocardial tissue was arranged regularly. In the MI group, the myocardium was replaced by a large piece of collagen tissue, and the remaining small amount of cardiomyocytes were disorderly arranged and the structure was blurred. The relative content of collagen in myocardial tissue in the MI group was significantly higher than that in the sham group. The cardiac fibrosis of the sham group and the MI group was described hereinbefore. The analysis of Masson staining suggested that, in the MI + MITF-NC group, cardiac tissues were replaced by massive collagen tissues, with granulation tissue hyperplasia observed. The microfibrillar collagen surrounding cardiomyocytes were broken, and disorderly aligned. The relative content of collage of cardiac tissues of the MI + MITF-NC group was similar to the MI group and significantly higher than the sham group (*P* < 0.05). The MI + MITF group showed evenly arranged cardiac tissues. Many cardiac tissues were replaced by collagen tissues, but the amount was smaller than the MI group (*P* < 0.05) (Figure 8A).

RETRACTED

**Figure 8:** **Upregulated MITF expression reduces cardiac fibrosis and promotes angiogenesis in MI rats.** (**A**) Masson staining showing the cardiac fibrosis of rats (× 200); (**B**) immunohistochemical staining showing the expression of type I collagen and type III collagen (× 200); (**C**) MVD and MMVD of cardiac tissues; (**D**) the mRNA expression of angiogenesis-related factor VEGF detected by RT-qPCR; (**E**) the protein expression of angiogenesis-related factor VEGF detected by western blot assay. * versus the sham group, *P* < 0.05; # versus the MI group, *P* < 0.05; n = 3. Data were analyzed by one-way ANOVA. Pairwise comparison after ANOVA was performed by Fisher’s least significant difference. MI, myocardial infarction; MITF, microphthalmia-associated transcription factor; MVD, microvascular density; MMVD, mean microvessels diameter; RT-qPCR, reverse transcription quantitative polymerase chain reaction; VEGF, vascular endothelial growth factor.

Immunohistochemical staining was used to observe the expression of type I collagen and type III collagen in cardiac tissues. Compared with the sham group, the MI and MI + MITF-NC groups manifested increased expression of type I collagen and type III collagen in cardiac tissues. Relative to the MI and MI + MITF-NC groups, the MI + MITF group showed decreased expression of type I collagen and type III collagen in cardiac tissues (*P* < 0.05) (Figure 8B).

The results of CD34 immunohistochemistry suggested that the MI rats had higher MVD than rats in the sham group. The MVD in the MI + MITF group was higher than the MI and MI + MITF-NC groups (*P* < 0.05). Additionally, relative to the sham group, the MMVD was decreased in the myocardial tissue of rats in the MI group, and the MMVD of rats in the MI + MITF group was greater than that of the MI group and the MI + MITF-NC group (both *P* < 0.05) (Figure 8C).

The RT-qPCR and western blot assay indicated that the mRNA and protein expression of VEGF in the MI + MITF group increased was significantly higher than that in the MI and MI + MITF-NC groups (*P* < 0.05) (Figure 8D–8E).

RETRACTED

### Upregulated MITF inhibits oxidative stress and inflammatory injury in rats with MI

The spectrocolorimetric method was employed to evaluate the levels of MDA and the activity of GSH-Px and SOD in cardiac tissues, so as to evaluate the effect of MITF on oxidative stress in MI rat models. Overexpressed MITF led to diminished serum levels of MDA and facilitated activity of GSH-Px and SOD (all *P* < 0.05) (Figure 9A).

**Figure 9:** **Upregulated MITF expression inhibits oxidative stress and inflammatory injury in MI rats.** (**A**) the levels of MDA and the activity of GSH-Px and SOD determined by the spectrocolorimetric method, n = 3; (**B**) the mRNA expression of IL-1β, IL-6 and TNF-α detected by RT-qPCR, n = 3; (**C**) the serum levels of IL-1β, IL-6 and TNF-α detected by ELISA, n = 6; * versus the sham group, *P* < 0.05; # versus the MI group, *P* < 0.05; Data were analyzed by one-way ANOVA. Pairwise comparison after ANOVA was performed by LSD-t. MI, myocardial infarction; MITF, microphthalmia-associated transcription factor; ELISA, enzyme-linked immunosorbent assay; IL-1β, interleukin-1β; IL-6, interleukin-6; TNF-α, tumor necrosis factor-α; MDA, malondialdehyde; GSH-Px, glutathione peroxidase; SOD, superoxide dismutase; RT-qPCR, reverse transcription quantitative polymerase chain reaction.

RT-qPCR and ELISA were performed to determine the mRNA and serum levels of IL-1β, IL-6 and TNF-α. Relative to the MI and MI + MITF-NC groups, the mRNA expression in cardiac tissues and serum levels of IL-1β, IL-6 and TNF-α were decreased in the MI + MITF group (all *P* < 0.05) (Figure 9B–9C), indicating that promoted MITF expression could ameliorate the oxidative stress and inflammatory injury of MI rats.

### Inhibited MITF expression reverses the improvement stimulated by miR-218 inhibitors for cardiac function and fibrosis in rats with MI

To verify whether miR-218 affects the cardiac function and fibrosis through negatively regulating MITF, we set the MI + miR-218 inhibitors + siRNA-MITF group, with the MI + miR-218 inhibitors + siRNA-NC group as a control. Relative to the MI + miR-218 inhibitors + siRNA-NC group, the MI + miR-218 inhibitors + siRNA-MITF group showed reduced cardiac function and decreased LVEF and LVFS (Figure 10A), increased LVEDP and reduced LVSP, +dp/dt max and -dp/dt max (Figure 10B), increased ratio of heart to body weight (Figure 10C), increased serum levels of LDH and CPK (Figure 10D), promoted pathological damages in cardiac tissues (Figure 10E–10F), enlarged infarct size (Figure 10G), elevated apoptotic index of cardiomyocytes (Figure 10H), increased Bax expression and reduced Bcl-2 expression in cardiac tissues (all *P* < 0.05) (Figure 10I).

RETRACTED

**Figure 10:** **The effect of downregulation of miR-218 and MITF on the cardiac function and fibrosis in MI rats. a refers to the MI + miR-218 inhibitors + siRNA-NC group and b refers to the MI + miR-218 inhibitors + siRNA-MITF group.** (**A**) the LVEF and LVFS of rats detected by ultrasonic cardiogram, n = 12; (**B**) the LVSP, LVEDP, +dp/dt max and -dp/dt max of rats detected by hemodynamic monitoring, n = 12; (**C**) the ratio of heart to body weight, n = 6; (**D**) serum levels of LDH and CPK examined by the biochemical analyzer, n = 6; (**E**) HE staining showing pathological changes of cardiac tissues (× 200), n = 3; (**F**) ultrastructure of cardiomyocytes observed by transmission electron microscope (× 5000), n = 3; (**G**) TTC staining showing the infarct size of rats, n = 3; (**H**) TUNEL staining showing the apoptotic index of cardiomyocytes (× 400), n = 3; (**I**) Western blot assay showing protein levels of apoptosis-related factors Bax and Bcl-2 in cardiac tissues, n = 3; (**J**) Masson staining showing the cardiac fibrosis of rats (× 200); (**K**) immunohistochemical staining showing the expression of type I collagen and type III collagen (× 200); (**L**) MVD and MMVD of cardiac tissues; (**M**) the mRNA and protein expression of angiogenesis-related factor VEGF detected by RT-qPCR and western blot assay; (**N**) the levels of MDA and the activity of GSH-Px and SOD determined by the spectrocolorimetric method, n = 3; (**O**) the mRNA expression of IL-1β, IL-6 and TNF-α detected by RT-qPCR, n = 3; (**P**) the serum levels of IL-1β, IL-6 and TNF-α detected by ELISA, n = 6; Data were analyzed by t test. MI, myocardial infarction; LVEF, left ventricular ejection fraction; LVFS, left ventricular fraction shortening; LVSP, left ventricular systolic pressure; LVEDP, left ventricular end diastolic pressure; RT-qPCR, reverse transcription quantitative polymerase chain reaction; MITF, microphthalmia-associated transcription factor; miR-218, microRNA-218; LDH, lactate dehydrogenase; CPK, creatine phosphokinase; MVD, microvascular density; MMVD, mean microvessels diameter; VEGF, vascular endothelial growth factor; ELISA, enzyme-linked immunosorbent assay; IL-1β, interleukin-1β; IL-6, interleukin-6; TNF-α, tumor necrosis factor-α; MDA, malondialdehyde; GSH-Px, glutathione peroxidase; SOD, superoxide dismutase.

The cardiac fibrosis was enhanced in MI rat models. Relative to the MI + miR-218 inhibitors + siRNA-NC group, the MI + miR-218 inhibitors + siRNA-MITF group had increased cardiac collagen (Figure 10J) and expression of type I collagen and type III collagen in cardiac tissues (Figure 10K).

RETRACTED

Angiogenesis was inhibited in MI rats. Versus the MI + miR-218 inhibitors + siRNA-NC group, the MI + miR-218 inhibitors + siRNA-MITF group displayed reduced MVD and MMVD (Figure 10L) and expression of VEGF mRNA and protein in cardiac tissues (all *P* < 0.05) (Figure 10M).

Oxidative stress and inflammatory injury were accelerated in MI rat models. the MI + miR-218 inhibitors + siRNA-MITF group showed increased MDA levels and reduced activity of GSH-Px and SOD (Figure 10N), increased mRNA expression and serum levels of IL-1β, IL-6 and TNF-α(all *P* < 0.05) (Figure 10O–10P).

These results indicated that inhibition of MITF expression could reverse the improvement induced by miR-218 inhibitors in cardiac function and fibrosis, confirming that miR-218 functioned in the cardiac function and fibrosis in MI rat models through inhibiting MITF expression.

## DISCUSSION

The chronic maladaptive process following MI as left ventricular remodeling is characterized by progressive cardiac fibrosis, myocardial hypertrophy, and deterioration of cardiac function over time, eventually leading to the occurrence of congestive heart failure [29]. Functional regulation of miRs has been hypothesized to reduce cardiomyocyte death and cardiac fibrosis following MI and improves the recovery of cardiac function [30]. For example, miR-21 [31] and miR-574-5p [32] are highly expressed in the settings of heart failure, and miR-29 [33] and miR-146a [34] are induced in the process of senescence of the heart. In this study, we identified induced miR-218 expression in rat models of MI and its association with cardiac fibrosis and cardiac function impairment through negative regulation of MITF.

MI leads to cardiac fibrosis and scar formation, which then results in loss of cardiomyocytes in the ischemic region of the heart, which reduces the contractility and deteriorate cardiac angiogenesis [35]. This study established MI models through left anterior descending coronary artery ligation in rats, after which, we observed cardiac function impairment, cardiomyocyte apoptosis, cardiac fibrosis, oxidative stress and inflammatory injury. Notably, higher expression levels of miR-218 and lower expression levels of MITF were determined in the cardiac tissues of MI rats. Studies have reported that miR-218 is down-regulated in multiple cancers and can act as a tumor suppressor by binding to and regulating different proteins [36, 37]. Yang et al. argues that miR-218 expression is associated with the activity of apocynin in mediating myocardial injury and fibrogenesis [38]. Another study reported by Fish et al. hypothesized that a Slit/miR-218/Robo regulatory loop is clearly required for the heart tube formation in zebrafish [20]. Expression of miR-218 was observed to be significantly increased in aortic endothelial cells of mice under intermittent hypoxia [39].

RETRACTED

Based on an initial bioinformatics prediction followed by a confirmatory dual-luciferase reporter gene assay, the targeting relationship between miR-218 and MITF was determined. MITF is a critical modulator of melanogenic enzymes in melanogenesis, and its expression is modulated by multiple transcriptional factors through miRs [27]. As a key transcriptional factor, MITF is targeted by many miRs expression profiles in melanocytes [40], for example, specific miRs, including miR-25, 182 and 204/211 [41–43]. Ectopic miR-218 could diminish the MITF expression and the inverse correlation was proved between MITF and miR-218 in human melanoma cells and primary skin melanocytes [27].

In the MI rat models, miR-218 inhibitors and/or MITF overexpression plasmid were injected into rats to investigate the effect of miR-218 and/or MITF on the cardiac function, pathological damage of cardiac tissues, cardiac fibrosis, angiogenesis, oxidative stress and inflammatory injury. The experimental results suggested that downregulated miR-218 and upregulated MITF improved cardiac function, alleviated pathological damage of cardiac tissues, reduced cardiac fibrosis, promoted angiogenesis, and reduced oxidative stress and inflammatory injury in MI rat models. A previous study has documented that inhibition of miR-218 could decrease expression of VEGF, caspase-3 and Bax and increase expression of Bcl-2 in aortic endothelial cells under intermittent hypoxia condition [39]. In cardiac myxoma, miR-218 could influence the cell proliferation of myxoma and the tumorigenicity through mediating the MEF2D expression by binding to the mRNA 3'UTR [44]. The involvement of miR-218 in cardiomyocyte hypertrophy has been indicated to act through binding to REST [45]. Moreover, downregulation of miR-218 can diminish the heart defects induced by overexpression of TBX5, leading to the notion that miR-218 is a candidate mediator of TBX5 in the heart development and possible association with the occurrence of heart malformations [19]. MITF is an anti-oxidant transcription factor, whose deficiency in mice leads to higher levels of reactive oxygen species and oxidative damage [46]. Thus, the treatment of overexpression plasmid of MITF could reduce oxidative stress following MI. More importantly, downregulation of MITF could reverse the rescue induced by miR-218 inhibitors in cardiac function and fibrosis, suggesting that miR-218 exerted function in the cardiac function and fibrosis in MI rat models through inhibiting MITF expression.

RETRACTED

Based on observations and evaluations made during the study, it was suggested that downregulated miR-218 improved cardiac function, alleviated pathological damage of cardiac tissues, reduced cardiac fibrosis and promoted angiogenesis, reduced oxidative stress and inflammatory injury in MI rat models through upregulating MITF expression. Currently, miR therapeutics are entering the stage as novel candidates for treatment of MI, but confirmed feasibility, toxicity profile and pharmacodynamics should be further investigated in future studies. Ultimately, this may go to the development of potential diagnostic and miR-based treatments for MI by diminishing cardiac fibrosis and function impairment.

## MATERIALS AND METHODS

### Experimental animals

Totally, 96 Sprague Dawley (SD) rats (weighing 280 ± 20 g) were purchased from Beijing Vital River Laboratory Animal Technology Co., Ltd. (Chaoyang district, Beijing, China). Prior to the experiments, the rats were raised to adapt to the new conditions for one week. The rats were housed in clean animal rooms with room temperature of 18-24°C, 12 h light/dark cycle and ad libitum to food and water. All experimental protocols used in this study were performed with the approval of the Ethics Committee for First Affiliated Hospital of Zhejiang University.

### Model establishment

Before model establishment, the rats were deprived of food for 12 h. The rats were anesthetized with 1% pentobarbital sodium (Sigma, Santa Clara, CA, USA). The skin was longitudinally cut open in the left side of the midline of the chest. The chest was opened at the position with the most obvious cardiac impulse to expose the heart. The anterior descending coronary artery was ligated by a suture 1 mm below the left atrial appendage through the space between the left atrial appendage and pulmonary conus. Immediately, the heart was reset and the chest was closed. Chest compressions were performed to resume spontaneous breathing. In the sham group, the coronary artery was threaded without ligation. During the week after the operation, the rats were injected intramuscularly with 800,000 U penicillin every day to resist infection. Ultrasonic cardiogram and hemodynamic monitoring were performed to identify whether model establishment was successful.

### Animal grouping

The rats were numbered according to the body weight and randomly classified into eight groups with 12 rats in each group: sham group, MI group, MI + inhibitors NC group (48 h before model establishment, NC of miR-218 inhibitors was injected into the caudal vein per day for two days), MI + miR-218 inhibitors group (48 h before model establishment, miR-218 inhibitors were injected into the caudal vein per day for two days), MI + MITF-NC group (48 h before model establishment, MITF-NC [NC of MITF overexpression plasmid] was injected into the caudal vein per day for two days), MI + MITF group (48 h before model establishment, MITF overexpression plasmid was injected into the caudal vein per day for two days), MI + miR-218 inhibitors + siRNA-NC group (48 h before model establishment, miR-218 inhibitors and siRNA-NC [NC of MITF interference plasmid] were injected into the caudal vein per day for two days), MI + miR-218 inhibitors + siRNA-MITF group (48 h before model establishment, miR-218 inhibitors and siRNA-MITF were injected into the caudal vein per day for two days). The inhibitors NC, miR-218 inhibitors, MITF-NC, MITF, siRNA-NC and siRNA-MITF plasmids were synthesized by Sangon Biotech Co., Ltd. (Shanghai, China).

RETRACTED

### Ultrasonic cardiogram

Two weeks after the model establishment, the rats were anesthetized and fixed in the supine position on the ultrasonic testing table. The probe was maintained steadily and transferred to M-mode to scan the cut surface with images captured. The left ventricular end-diastolic volume (LVEDV) and left ventricular end systolic volume (LVESV) were determined in order to calculate the left ventricular ejection fraction (LVEF) and left ventricular fraction shortening (LVFS): LVEF (%) = (LVEDV - LVESV) / (LVEDV) × 100%.

### Hemodynamic monitoring

After the examination of ultrasonic cardiogram, the neck tissues were isolated bluntly to expose the carotid artery. Then the carotid artery was ligated at the distal end and pulled by a thread at the proximal end. A 1.4 F Millar catheter was inserted into the carotid artery. When the Millar catheter went into the left ventricular, the left ventricular end diastolic pressure (LVEDP) and maximum rate of rise of left ventricular pressure increase (+dp/dt max) and the maximum rate of rise of left ventricular pressure decrease (-dp/dt max) were examined. Whether the catheter was inserted into the left ventricular was determined according to the pressure waves.

### Specimen collection and indicator detection

After the hemodynamic monitoring, six rats were taken from each group, with body weight weighed. The abdomen was opened, and blood was collected through the aorta abdominalis. The blood was centrifuged at 1500 r/m for 10 min, with supernatant stored in a refrigerator at −70°C to detect indicators in serum. The heart was extracted and weighted after the heart was opened to calculate the ratio of the heart to total body weight. The cardiac tissues of three rats were extracted for hematoxylin-eosin (HE) staining, Masson staining, immunohistochemistry and terminal deoxyribonucleotidyl transferase (TDT)-mediated dUTP-digoxigenin nick end labeling (TUNEL) staining. The cardiac tissues of remaining three rats were immersed in liquid nitrogen and stored in a refrigerator at −80°C for detection of indicators of oxidative stress, reverse transcription quantitative polymerase chain reaction (RT-qPCR) and western blot assay.

RETRACTED

The spectrocolorimetric method was adopted to examine the levels of oxidative stress indicators including malondialdehyde (MDA), glutathione peroxidase (GSH-Px) and superoxide dismutase (SOD) (Nanjing Jiancheng Bioengineering Institute, Nanjing, Jiangsu, China) in the tissue homogenate.

A MODULAR-DPP automatic biochemical analyzer (Roche, Basel, Switzerland) was employed to determine the levels of lactate dehydrogenase (LDH) and creatine phosphokinase (CPK) in serum.

Enzyme-linked immunosorbent assay (ELISA) was performed to determine the serum levels of interleukin-1β (IL-1β), interleukin-6 (IL-6) and tumor necrosis factor-α (TNF-α) (Nanjing Jiancheng Bioengineering Institute, Nanjing, Jiangsu, China).

### HE staining

The hearts of three rats were cut off from the root of aorta and immediately placed in the precooled phosphate-buffered saline (PBS) at 4°C to rinse the blood. The hearts were fixed in paraformaldehyde for 24 h. Then the hearts were embedded in paraffin to prepare tissue blocks, which were sliced to sections with a thickness of 5 μm. Following HE staining, the sections were observed and photographed under an optical microscope, in order to observe the staining distribution and intensity of the cardiac tissues.

### Masson staining

Three sections of cardiac tissues were taken from each rat of each group. After Masson staining, the cardiomyocytes were presented with red color under the optical microscope, and collagenous fibers with blue-green color. Image-Pro plus 6.0 software (Media Cybernetics, Rockville, Maryland, USA) was used for quantitative analysis of the collagen volume fraction (CVF = collagen area of the same image / the detected field area) for each field of sections. The vessels and scar region with abundant collagen were excluded. Five fields were selected for each section with average value calculated.

### Immunohistochemistry

Three sections of cardiac tissues were taken from each rat of each group. Endogenous peroxidase activity was quenched with 3% hydrogen peroxide. Antigen retrieval was performed by 0.1 mol/L citric acid buffer for 20 min, followed by blocking in 10% rabbit serum for 30 min. Primary antibodies to type I collagen, type III collagen and CD34 (1: 50) working solution were added, followed by incubation at 4°C for 16 h. The horseradish peroxidase-labeled goat anti-rat secondary antibody was added for incubation at room temperature for 2 h, followed by diaminobenzidine development. The protein expression conditions were observed and photographed under an optical microscope. Image-Pro plus 6.0 image software was adopted. Five fields were randomly selected for each section. The integrated optical density (IOD) was analyzed after determining the grey value of immunohistochemical images. The IOD was regarded as the quantitative expression of type I collagen and type III collagen, with brown color as positive expression. The staining of CD34 antibody demonstrated the microvascular density (MVD). After immunohistochemical staining with CD34 polyclonal antibody, vascular endothelial cells were stained as brownish yellow granules. According to the method of Weidner et al. [47], the infarct area was firstly imaged under a low magnification, and then the brown cells and cell clusters were observed under a high magnification (200 times, 400 times). Where brown single endothelial cells or endothelial cell clusters appeared as a blood vessel count, and blood vessels with a lumen greater than 50 um were not counted, and five vessels with the highest vessel density under the 400 times microscope were selected for microvessel count, and then the average value was calculated as a sample of MVD. For CD34 staining sections, two samples of 400-fold field of view were randomly selected for each sample. The length of the short axis of the blood vessel was measured by Image-ProPlus 6.0 software, and the average value was calculated as the mean microvessels diameter (MMVD).

RETRACTED

### TUNEL staining

Three sections of cardiac tissues were taken from each rat of each group. According to the instructions of TUNEL apoptosis kit (Thermo Fisher Scientific, Waltham, MA, USA), TUNEL staining was performed. After staining, the specimens were magnified 400 ×. The positive cells were brownish yellow. The fields in the infarct area and surrounding areas were randomly selected. The percentage of apoptotic cells in total cells was regarded as the apoptotic index of cardiomyocytes.

### Transmission electron microscope (TEM) observation

After the hemodynamic monitoring, three rats of each group were euthanatized by cervical dislocation with the heart extracted. About 1 mm^3^ left ventricular was cut and fixed in 1% osmic acid and then in 2.5% glutaraldehyde. The left ventricular was dehydrated gradiently in acetone, embedded in Epon 812 epoxy resin and sliced by a ultrathin slicer. The sections were stained by 1% uranyl acetate-lead citrate. The ultrastructure of cardiomyocytes was observed under the TEM.

### 2,3,5-triphenyltetrazolium chloride (TTC) staining

After the hemodynamic monitoring, the remaining three rats were anesthetized and their chests were opened. The freshly prepared 1% TTC solution (1 mL, Sigma, Santa Clara, CA, USA) was slowly injected through the inferior vena cava and the heart was allowed to beat for 3~4 min. Following this, the heart was extracted and the remaining bloodstain was rinsed by normal saline. Then the heart was immediately frozen for 10 min at -80°C and sliced to sections. The sections were fixed in 4% paraformaldehyde for 20~30 min. The staining images were captured by a digital camera and analyzed by the Image-Pro plus 6.0 software. The area of white region (infarct region) and left ventricular region were measured to calculate the myocardial infarct area = area of infarct region / area of left ventricular region × 100%.

RETRACTED

### RT-qPCR

Trizol method (Invitrogen, Carlsbad, CA, USA) was adopted to extract total RNA of cardiac tissues. The high quality of RNA was confirmed by ultra-violet analysis and formaldehyde gel electrophoresis. RNA (1 μg) was collected and avian myeloblastosis virus reverse transcriptases were employed for reverse transcription to get cDNA. The primers of PCR were designed and synthesized in Invitrogen (Carlsbad, CA, USA) (Table 1). Glyceraldehyde-3-phosphate dehydrogenase (GAPDH) was regarded as an internal reference of target genes and U6 as the internal reference of miR-218. The amplification conditions were pre-denaturation at 94°C for 5 min, denaturation at 94°C for 40 s, annealing for 40 s at 60°C, DNA strands extension for 1 min at 72°C, this protocol ran for 40 cycles, followed by extension for 10 min (72°C). The PCR products were verified by agarose gel electrophoresis. Threshold value was manually selected at inflection point of all parallel rising logarithmic amplification curves, and the threshold cycle (Ct) value of each reaction tube was recorded. The data were analyzed by 2^-ΔΔCt^ method, which represents the ratio of gene expression of the experimental group to the control group. The formula was ΔΔCt = [ΔCt _target gene_ - ΔCt _reference gene_]_experimental group_ - [ΔCt _target gene_ - ΔCt _reference gene_]_control group_. The experiment was conducted in triplicate with mean value calculated.

**Table 1:** Primer sequences for reverse transcription quantitative polymerase chain reaction.

**Gene**	**Primer sequence**
miR-218	F: 5′- GCGCTTGT-GCTTGATCTAA -3′
	R: 5′- GTGCAGGG-TC-CGAGGT -3′
U6	F: 5′-CGCTTCGGCAGCACATATAC-3′
	R: 5′- AAATATGGAACGCT-TCACGA -3′
MITF	F: 5′- GAGAGAGCAGGACACCATCG -3′
	R: 5′- GCACAAACTTGCCACAGTGT -3′
VEGF	F: 5′- TTGTCTCAGGCAGAAGTCC -3′
	R: 5′- CAAAGAAACGCCACCATT -3′
IL-1β	F: 5′- GAAGGCAGTGTCACTCATT -3′
	R: 5′- TCTTTGGGTATTGTTTGG-3′
IL-6	F: 5′- AGCCCACCAGGAACGAAAG -3′
	R: 5′- GGAAGGCAGTGGCTGTCAA -3′
TNF-α	F: 5′- CTGTGAAGGGAATGGGTGTT -3′
	R: 5′- GGGCTGGCTCTGTGAGGAAG -3′
GAPDH	F: 5′- ACGGCAAGTTCAACGGCACAG -3′
	R: 5′- GACGCCAGTAGACTCCACGACA -3′

Note: miR-218, microRNA-218; F, forward; R, reverse; GAPDH, glyceraldehyde-3-phosphate dehydrogenase; MITF, microphthalmia-associated transcription factor; VEGF, vascular endothelial growth factor; IL-1β, interleukin-1β; IL-6, interleukin-6; TNF-α, tumor necrosis factor-α.

RETRACTED

### Western blot assay

The protein of cardiac tissues was extracted, with protein concentration determined according to the bicinchoninic acid (BCA) protein assay kit (Wuhan Boster Biological Technology Co., Ltd., Wuhan, Hubei, China). The extracted protein with uploading buffer was boiled at 95°C for 10 min, 30 μg sample was uploaded for each well. Then, 10% polyacrylamide gel electrophoresis was employed to separate proteins, with electrophoresis voltage 80 V transferring to 120 V by wet transfer. The proteins were transferred onto polyvinylidene fluoride membranes with transferring voltage of 100 mV for 45-70 min. The membranes were blocked with 5% bovine serum albumin for 1 h. Primary antibodies to MITF, vascular endothelial growth factor (VEGF), Bcl-2 and Bax (1 : 1000) and β-actin (1 : 3000) (ab20663, ab46154, ab196495, ab53154 and ab227387, Abcam, Cambridge, MA, USA) were added and incubated at 4°C overnight, followed by washing three times (5 min per wash) with Tris-buffered saline with Tween 20 (TBST). Corresponding secondary antibodies (Shanghai Miaotong Biotechnology Co., Ltd., Shanghai, China) were added and incubated for 1 h. The membranes were washed for three times (5 min per wash). Chemiluminescence reagents were employed to develop images. β-actin was used as an internal reference. The images of the gels were captured in a Gel Doc EZ Imager (Bio-Rad, Hercules, CA, USA). The grey values of target protein bands were analyzed by ImageJ software (National Institutes of Health, Bethesda, Maryland, USA). The experiment was conducted in triplicate with mean value calculated.

### Dual-luciferase reporter gene assay

The bioinformatics website (http://www.targetscan.org) was adopted to predict the targeting relationship between miR-218 and MITF and binding sites of miR-218 to MITF. MITF 3′untranslated region (UTR) promoter sequence containing miR-218 binding sites were synthesized. MITF-3′UTR-wild type (WT) plasmid was constructed. According to this plasmid, binding sites were mutated to construct MITF-3′UTR-mutant type (MUT) plasmid based on the instructions of plasmid extraction kit (Promega Corporation, Madison, WI, USA). Cells at logarithmic growth phase were inoculated in the 96-well plate. When cell confluence reached 70%, transfection was performed based on the instructions of Lipofectamine 2000 (Invitrogen, Carlsbad, CA, USA). MITF-3′UTR-WT and MITF-3′UTR-MUT plasmids were mixed with miR-218 mimics and mimics NC were co-transfected into the 293T cells. The miR-218 mimics and mimics NC were purchased from Sangon Biotech Co., Ltd. (Shanghai, China). After transfection of 48 h, cells were harvested and lysed. The luciferase activity was determined by using a dual-luciferase reporter gene assay kit (BioVision, San Francisco, CA, USA). The experiment was conducted in triplicate.

RETRACTED

### Statistical analysis

SPSS 21.0 (IBM-SPSS Corp, Armonk, NY, USA) was employed to analyze data. The data were confirmed with normal distribution after Kolmogorov-Smirnov test. The results were presented by mean ± standard deviation. Data between two groups were analyzed by *t* test. Comparison among multiple groups was analyzed by one-way analysis of variance (ANOVA), after which pairwise comparison was conducted by the Fisher’s least significant difference t test (LSD-t). The two-tailed test was considered significant if *P* < 0.05.
